# Application of the Preoperative Assistant System Based on Machine Learning in Hepatocellular Carcinoma Resection

**DOI:** 10.1155/2021/4757668

**Published:** 2021-09-24

**Authors:** Shouyun Lv, Shizong Li, Zhiwei Yu, Kaiqiong Wang, Xin Qiao, Dongwei Gong, Changxiong Wu

**Affiliations:** ^1^Occupational Health Department, Haikou Center for Disease Control & Prevention, Haikou 571101, China; ^2^Hepatobiliary and Pancreatic Surgery, Hainan General Hospital, Haikou 570311, China

## Abstract

To conduct better research in hepatocellular carcinoma resection, this paper used 3D machine learning and logistic regression algorithm to study the preoperative assistance of patients undergoing hepatectomy. In this study, the logistic regression model was analyzed to find the influencing factors for the survival and recurrence of patients. The clinical data of 50 HCC patients who underwent extensive hepatectomy (≥4 segments of the liver) admitted to our hospital from June 2020 to December 2020 were selected to calculate the liver volume, simulated surgical resection volume, residual liver volume, surgical margin, etc. The results showed that the simulated liver volume of 50 patients was 845.2 + 285.5 mL, and the actual liver volume of 50 patients was 826.3 ± 268.1 mL, and there was no significant difference between the two groups (*t* = 0.425; *P* > 0.05). Compared with the logistic regression model, the machine learning method has a better prediction effect, but the logistic regression model has better interpretability. The analysis of the relationship between the liver tumour and hepatic vessels in practical problems has specific clinical application value for accurately evaluating the volume of liver resection and surgical margin.

## 1. Introduction

Hepatectomy is one of the main methods of surgical treatment of liver cancer, such as hepatitis B, liver cirrhosis, and the application of surgical resection is limited. Too much resection of the liver may cause severe postoperative liver dysfunction, so the remaining liver volume is over 30%; for patients with liver cirrhosis, the remaining liver volume exceeds 50% to prevent postoperative liver failure [1]. Therefore, it is essential to accurately evaluate the liver condition before surgery, which mainly relied on CT examination in the past. In 2008, Intrasense developed Myrian XP-Liver, a new three-dimensional surgical simulation system that automates liver segmentation and performs virtual surgery, simultaneously calculating liver volume for preoperative evaluation and surgical simulation. This study used this software to perform preoperative assessment and surgical simulation of patients undergoing precision hepatectomy. The simulated data were compared with the actual situation during the operation to evaluate the application value of the three-dimensional surgical simulation system in precision hepatectomy [2].

Hepatectomy is an effective treatment for liver cancer, hilar cholangiocarcinoma (and benign liver tumors), hepatolithiasis, and other liver diseases. Since the beginning of the twenty-first century, under the guidance of the concept of precision medicine, supported by functional liver anatomy, pathological anatomy, new imaging technologies, new methods of liver function evaluation, and new technologies of liver parenchyma separation, precision liver resection has become the forefront of liver surgery [3]. It is developing new strategies for early prediction of cancer treatment based on machine learning methods. Logistic regression, random forest, support vector machine, C5.0 decision tree, neural network, bagging algorithm, and AdaBoost algorithm were used to construct the three-year tumour-free survival time (disease-free survival, DFS). The classification and extraction rules of clinical medical data of liver tumours are extracted through the three-year overall survival (OS) model to achieve early prediction and assist clinical diagnosis [4–6]. It fulfils early prediction and early treatment, and improves the survival rate of patients with liver tumours. Since the beginning of the 21st century, under the guidance of the concept of precision medicine, supported by new methods of functional liver anatomy, pathological anatomy, imaging, liver function evaluation, and modern liver parenchyma separation technology, precision hepatectomy has become a cutting-edge technology in liver surgery. Based on segmented liver resection, this surgical method strives to remove the lesion altogether while achieving “minimum trauma, maximum organ protection, and best rehabilitation effect,” which embodies the fundamental transformation of the patient-centred medical model.

Modern surgical procedures in the twenty-first century have made the pure pursuit of surgical curative effects a temporary thing [7–9]. In the field of surgery, every innovation cannot be separated from the development and progress of imaging technology. The emergence of CT and MRI has had a far-reaching impact on surgery and even the whole medical area. The ability to “see” gives surgeons an ideal space for display [10]. New imaging technology, which requires not only “seeing clearly” but also “seeing well” and has the function of virtual operation, has become another essential technical demand in the field of liver surgery in the new era [11]. Relying on the development of digital imaging technology, three-dimensional accurate surgical planning system has developed vigorously in the medical field in recent years. With the help of traditional two-dimensional visual data imaging technology, three-dimensional accurate surgical planning system can carry out high-resolution digital three-dimensional reconstruction according to the needs of surgeons and rotate, move, or zoom the three-dimensional model in an all-round way. At the same time, you can also select various organs, blood vessels, nerves, and diseased tissues, adjust the transparency and color of each organ model, and perform three-dimensional spatial data measurement. The surgeon forms a traditional two-dimensional image to reconstruct the virtual 3D image and move it to the screen for a more intuitive understanding of the lesion and its surrounding anatomy [12–14].

According to reports, the application of the surgical planning system in liver surgery has developed to a certain extent. Compared with the traditional two-dimensional image data, the 3D surgical planning system can determine the location of the lesion, accurately distribute the liver blood vessel structure, and improve the accuracy of liver surgery. And simulated surgery, the assessment of residual liver volume has its unique characteristics. However, does this mean that we can completely trust the results and ignore the clinical experience and surgeon's surgical techniques [15]? This study included the INCOOL3D precision surgery planning analysis system of the Department of Hepatobiliary and Pancreatic Surgery of Wuhan Central Hospital to plan prehepatectomy. This article analyzes clinical data, compares the application of the surgical planning system and traditional imaging data in the application of liver surgery, and evaluates the application of the liver resection surgery planning system application value. The deficiencies found in the operation planning system were illustrated with examples, and the reasons were analyzed. The application of the operation planning system and intraoperative ultrasound in hepatectomy was compared. It is expected to provide some guidance for the clinical application of a 3D surgical planning system.

## 2. Research Methods

### 2.1. Clinical Data

In this study, 50 patients who underwent precision hepatectomy for liver cancer in the Department of Hepatobiliary Surgery of the First Affiliated Hospital of Sun Yat-sen University from June to December 2020 were selected as the research objects, including 30 males and 20 females, with an average age of 50 years. The patient had a precise diagnosis of liver cancer (AFP > 400 *μ*g/L and positive for one or more dynamic imaging tests) and no contraindication to surgery [16–18]. There were no patients with postoperative recurrence and planned reoperation. The tumour diameter ranged from 1.5 to 20.5 cm (9.6 ± 4.9 cm). The Child-Pugh grade of liver function before surgery was A/B; the retention rate of indole green for 15 min (ICG15 min) was less than 10%. The AFP was 1–58,344 *μ*g/L (7,782.7 ± 17,573.9 *μ*g/L). There were 13 cases of tumours adjacent to important tissue structure (portal vein, inferior vena cava, hepatic vein, diaphragm, and right adrenal gland). There were 7 cases of vascular tumour thrombus formation, including four circumstances of portal vein tumour thrombus and one case of hepatic vein tumour thrombus.

#### 2.1.1. Logistic Regression Model

Logistic regression makes statistical inference and data analysis through hypothesis test, which is mainly applicable to risk factor analysis of epidemiological data, clinical trial evaluation, and prognostic factor analysis of diseases. The regression coefficients of each variable were calculated to screen the variables and establish a regression model [19]. The study in this paper is about whether patients with liver tumour relapse or survival within three years, which is a dichotomy problem. Logistic forward stepwise regression analysis was used for feature selection, and a logistic regression prediction model was established to obtain the prognosis models of three-year tumour-free survival and overall survival.

#### 2.1.2. Random Forest

Random forest is a tree-shaped set of classifiers in which the metaclassifier uses the CART algorithm. X is the input vector, a random vector of the independent branch library, which determines the growth process of a single tree. Random forest uses the self-service method (bootstrap resampling technology) to rewind from the original *N* training sample set and repeat *k* random samples to generate a new training sample set and then generate *k* random self-service classification tree forests based on the sample set. The latest data is classified. The result is based on the classification tree to vote for multiple forms of scores [20]. In essence, it is an improvement of the decision tree algorithm. Numerous decision trees are merged, and the establishment of each tree depends on an independent sample. Each tree in the forest has the same distribution, and the classification error depends on the classification ability of each tree and the correlation between them.

The basic model of the support vector machine (SVM) is to find the best separation hyperplane in the feature space to maximize the interval between positive and negative samples on the training set $D=\left\{\left(\overset{⟶}{x_{1}}y_{1}\right),\left(\overset{⟶}{x_{2}}y_{2}\right),\ldots \left(\overset{⟶}{x_{n}}y_{n}\right),\right\},y_{i}\in \left\{+1-1\right\}$. Given a training sample set, *I* represents the *i*th sample, and *n* represents the sample size.

The following linear equation can describe the hyperplane:

(1) $$\begin{array}{c} {\overset{⟶}{\omega }}^{T}\overset{⟶}{x}+b=0, \end{array}$$

where the representation vector $\overset{⟶}{\omega }$ determines the direction of the hyperplane and *B* represents the offset, which determines the distance between the hyperplane and the origin. The optimal hyperplane is found for hypothesis *D* of the training data set $\overset{⟶}{\omega }*\overset{⟶}{x}+b^{*}=0$, and the decision classification function is defined as follows:

(2) $$\begin{array}{c} f\left(\overset{⟶}{x}\right)=\text{sign}\left({\overset{⟶}{\omega }}^{*}\overset{⟶}{x}+b^{*}\right). \end{array}$$

### 2.2. CT Examination and 3D Reconstruction

The patients were routinely examined preoperatively with enhanced CT using Toshiba 64-slice spiral CT with an interlayer interval of 2 mm. The contrast agent was intravenously injected with iopromide (90 ml), and the CT data after phase III imaging were imported into the three-dimensional surgical planning system. When the liver is segmented in semiautomatic mode, the 3D operator simulation system (Myrian XP liver) can automatically segment all normal liver and lesion areas by 3D reconstruction on the basis of CT scanning horizontal data of normal and pathological tissues, in every 4-5 times when necessary to manually tag scanning level to ensure the reconstruction accuracy. The same method can be used to reconstruct the blood vessels in the liver. The system also has virtual surgery, which can simulate the operation by setting different cutting planes and cutting lines to adjust the operational plan in time. During the whole process, the data of tumour volume, liver volume, residual liver volume, and surgical margin can be calculated using the software.

### 2.3. Precise Liver Resection

The Treitz ligament was separated, and the pedicle of the liver was exposed through a “human” incision. The liver parenchyma was isolated with an ultrasonic suction knife (CUSA knife) to tell the Glisson sheath of the hepatic segment or subsegment. The supplying blood vessels in the tumour-bearing hepatic segment were clamped with vascular forceps. The boundary of the ischemic area was marked on the surface of the liver with an electric knife. The vascular forceps were removed, and the supplying blood vessels in the hepatic segment were lifted with a rubber band. The portal vein branch of the corresponding hepatic segment was punctured with a 21-size fine needle; methylene blue (4 ml for each hepatic segment) was injected; and the pedicle of the corresponding hepatic segment was ligated after needle extraction. The actual extent of the liver segment was determined by the methylene blue staining range of liver parenchyma. Habib·4X bipolar device (Habib 4X bipolar resection device) was used to remove the liver segment where the tumour was.

### 2.4. Evaluation of the Accuracy of the Three-Dimensional Surgical Planning System

The software's accuracy was evaluated by comparing the simulated resected liver volume with the actual resected liver volume and the simulated surgical margin with the actual surgical margin of 50 patients. The resected liver was weighed by electronic scale, and the volume of 1 g liver was considered 1 ml. The distance between the surgical margin and the tumour was measured with callipers on the excised specimens, and the actual value and the simulated data were statistically analyzed.

### 2.5. Statistical Methods

SPSS13.0 software was used for statistical analysis. Data were expressed as mean ± standard deviation ([Akx-d]±*s*). The comparison of the actual value of surgical resection volume and surgical margin with the simulated value was performed by *t*-test. The correlation analysis between the actual value and the simulated value was performed by Pearson correlation analysis. The test level *α* is equal to 0.05.

## 3. Research Results

According to the preoperative surgical plan results combined with intraoperative ultrasound and actual surgical results and surgical methods, six cases of actual surgery were the same as the preoperative plan in four cases. One case was found to have severe liver cirrhosis during the operation, and the liver segment was removed after liver failure. There is a high risk of bleeding. Considering patients with liver tumours less than 2 cm in diameter, there is no significant difference in radiofrequency ablation and surgical resection efficacy. It has little effect on liver function. Radiofrequency ablation of the S3 tumour was performed after obtaining the consent of the patient's family members. In another case, intraoperative ultrasound showed multiple nodular lesions in the liver, but the preoperative CT scan and 3D surgical planning system did not show related lesions. According to the results of the intraoperative ultrasound, the possibility of malignant lesions could not be ruled out. Therefore, a total of 10 nodular lesions in the liver were performed radiofrequency ablation while resectioning S6 and S7 segments. Virtual hepatectomy was performed in the experimental group, and the volume of resected liver and residual liver were automatically calculated. The volume of resected specimens was measured after surgery and compared with the actual resected liver volume before surgery. There was no statistical difference between preoperative planning results (637.97 ± 817.18 ml) and actual postoperative resection results (618.40 ± 766.83 ml; *P* = 0.957 and *P* > 0.05). In the experimental group, six vessels were invaded, and six vessels were shown by the preoperative surgical planning system, with a coincidence rate of 100%. In the control group, seven vessels were confirmed by operation, and four vessels were confirmed by preoperative CT, with a coincidence rate of 57.1%. There was no statistical difference in preoperative vascular invasion between the experimental and control groups (*P* = 0.067).

### 3.1. Statistical Analysis between the Experimental Group and the Control Group

There were no significant differences in gender (*P* = 0.536), age ((53 ± 11.8)/(54.73 ± 8.65; *P* = 0.692), and surgical method (*P* = 0.611) between the experimental group and the control group (*P* > 0.05) as shown in Table 1. There were significant differences in operative time ((204.55 ± 46.55)/(247.27 ± 51.79; *P* = 0.015) and intraoperative blood loss ((199.09 ± 74.89)/(261.82 ± 60.63); *P* = 0.044) between the experimental group and the control group (*P* < 0.05). The operative time in the experimental group was shorter than that in the control group, and the amount of intraoperative bleeding in the experimental group was less than that in the control group. There were no significant differences between the experimental group and the control group in postoperative complications (*P* = 0.534) and length of hospital stay ((12.73 ± 2.49 d)/(12.18 ± 2.18 d); *P* = 0.591 and *P* > 0.05). In experimental group, multiple small nodules in the liver were accidentally found by intraoperative ultrasound, but preoperative CT and surgical planning system found no corresponding lesions. In the control group, three cases were found unexpected small lesions by intraoperative ultrasound but not by preoperative CT examination. Overall, in detecting small intrahepatic lesions, intraoperative ultrasound was evident due to CT examination and surgical planning systems.

### 3.2. Accuracy of the 3D Surgical Simulation System in the Simulation of Liver Volume and Surgical Margin

The liver volume and surgical margin of 50 patients were simulated preoperatively and compared with the actual postoperative volume and surgical margin. The results showed that there was a significant correlation between simulation and actual hepatectomy volume (*r* = 0.960, *P* < 0.001; Figure 1(a)), and there was no statistically significant difference between the mean values (896.7 vs. 819.1 ml; *t* = 1.851, *P* = 0.068). There was also a significant correlation between simulated and actual surgical margins (*r* = 0.972, *P* < 0.001; Figure 1(b)), and there was no statistical significance in the mean value (12.2 vs. 11.9 mm; *t* = 1.143, *P* = 0.256).

It can be seen from Tables 2 and 3 that the test set has better results than the training set.

For liver surgery, the traditional preoperative evaluation relies on two-dimensional CT findings. The surgeon evaluates the patient's condition according to his/her own experience. Only the doctor with rich clinical and radiograph reading experience can make a near-correct judgment on the patient's condition. The 3D surgical simulation software used in this study can integrate and reconstruct 2D CT data to form visual 3D images and calculate the volume and length of the region of interest, which plays an essential auxiliary role in surgeons' accurate understanding of patients' conditions before surgery and formulation of the appropriate surgical plan. This study uses three-dimensional operation simulation software for the whole liver volume, resection of liver volume, and residual liver volume calculation of automatic simulation of cutting a statistical correlation of liver volume and the actual results. Simulation results, on average, are more significant than the actual volume of 75.6 ml. Other 3D software calculations of 53.0 and 64.9 ml compared to larger, using 3D operation simulation in this study The software measured the distance between the surgical margin. The results showed that the simulated data were statistically correlated with the actual value. The mean difference between the simulated data and the actual value was 0.3 mm (12.2 vs. 11.9 mm), significantly smaller than previous reports. Therefore, the three-dimensional surgical simulation software has essential reference significance for accurate liver resection preoperative planning. By accurately predicting the surgical margin, an appropriate surgical resection range can be established to reduce the recurrence of postoperative liver cancer.

## 4. Conclusions

The 3D surgical simulation software collects information from 64-slice spiral CT with thin scanning layers, providing detailed information that traditional CT cannot provide. The whole reconstruction process was less than 30 min. The reconstructed image can clearly show the distribution of blood vessels in the Liver. There may be variation in intrahepatic vessels, whether hepatic artery, hepatic vein, or portal vein, so it is of great significance to accurately understand the anatomical relationship between tumour and blood vessel before surgery. Using various auxiliary functions of the software, surgeons can accurately understand the complex anatomy of the liver before the operation and simulate the possible conditions during the operation to adjust the surgical plan in time. In this study, the patient with a massive tumour of the right liver planned to undergo standard right hemihepatectomy. However, after preoperative simulation, the residual liver volume was less than 30% of the whole liver, and the possibility of liver failure was higher after surgery. Therefore, the surgical plan was adjusted, and the right hemihepatectomy with VIII segment reserved was changed to ensure that the residual liver volume exceeded 30% of the whole liver. No liver failure occurred after surgery, and the patient was cured and discharged from the hospital. In conclusion, the 3D surgical simulation software can accurately perform image reconstruction and volume calculation, and the virtual surgical function can assist surgeons in making surgical plans. The clinical application of this software has a specific auxiliary effect on the development of precision liver resection.

## Figures and Tables

**Figure 1:** Correlation analysis between simulated surgical indexes and actual surgical indexes: (a) volume of liver resection and (b) surgical margin.

**Table 1:** Comparison of data between the experimental group and control group.

	The experimental group, *N* = 10	The control group, *N* = 10	*P* ^*∗*^
Gender (M/F)	4 (40%)/6 (60%)	5.5 (55%)/4.5 (45%)	0.54
Age (y)	55	55	0.69
Operation method^*∗*^	1 (10%)/9 (90%)	3 (30%)/7 (70%)	0.61
Operation time (min)	205	245	0.02
Bleeding (ml)	200	260	0.04
Complications	1/10	2/10	0.56
Length of time (d)	15	12	0.60

**Table 2:** Predicting accuracy and AUC of each machine learning method.

Projects	Training set		Test set	
	Error rate	AUC	Error rate	AUC
Logistic regression	0.25	0.73	0.28	0.70
Random forest	0.16	0.83	0.28	0.71
SVM	0.26	0.73	0.28	0.71
C5.0 decision tree	0.24	0.74	0.28	0.70
Neural network	0.22	0.76	0.31	0.67
Bagging algorithm	0.24	0.73	0.29	0.69
AdaBoost algorithm	0.24	0.75	0.30	0.69

**Table 3:** Accuracy and AUC of tumour-free survival time of each machine learning method.

Projects	Training set		Test set	
	Error rate	AUC	Error rate	AUC
Logistic regression	0.22	0.70	0.25	0.67
Random forest	0.15	0.78	0.26	0.65
SVM	0.22	0.68	0.24	0.65
C5.0 decision tree	0.22	0.70	0.26	0.64
Neural network	0.20	0.71	0.28	0.62
Bagging algorithm	0.22	0.68	0.26	0.63
AdaBoost algorithm	0.15	0.78	0.26	0.65

## Data Availability

The data used to support the findings of this study are available from the corresponding author upon request.
